The article "Meta-Analysis of Children's Acute Psychological Stress and Action Stress on Immune Function under Microscope Images" was retracted in 2023. Reasons: unreliable results or conclusions; concerns about the data; concerns about the peer review; concerns about the citations.

# Meta-Analysis of Children's Acute Psychological Stress and Action Stress on Immune Function under Microscope Images

**DOI:** 10.1155/2022/6549805

**Published:** 2022-03-23

**Authors:** Hanjiang He, Yulin Tan, Lihua Li

**Affiliations:** ^1^School of Medicine, Lishui University, Lishui 323000, Zhejiang, China; ^2^School of Basic Medicine, Xiangnan University, Chenzhou 423000, Hunan, China

## Abstract

The immune system is a complex system, mainly including immune cells and immune organs. When the human body is invaded by foreign substances, the immune system will play a role in resisting the attack of harmful substances and pure necrotic cells, which is the defense structure of the body. The purpose of this study was to analyze children's acute psychological stress and action stress, and judge the adverse effects on immune function. Through the stress experiment of rats, three experimental groups were set up, which were placebo control group, placebo stress group, and drug stress group. The experiments include material-level test, sugar preference test, body weight test, and lymphocyte test. The experimental data show that stress reaction not only causes negative emotions, but also reduces weight gain by about 5%, and sugar preference decreases by about 40% compared with the normal group. There was no significant difference in the number of granulocytes and intermediate cells in the blood, but the number of lymphocytes increased from 2.49 × 10^9^/L to 5.03 × 10^9^/L. It shows that acute psychological stress has an inhibitory effect on the immune function of the body; not only suitable load exercise can improve the immune function of the body but also the mechanism may be that moderate load exercise makes the rat axis has better adaptability, and improves hormones, cytokines, and cytokines. The secretion of neurotransmitters can maintain the stability of the body's immune function.

## 1. Introduction

### 1.1. Background and Significance

Today, the public health problems widely studied are anxiety and depression, which are closely related to the prevention and treatment of post-traumatic anxiety disorder. Long-term or short-term strong fear may exceed the individual's ability to adapt and tolerate, causing changes in the body's nervous system, cardiovascular system, immune system, endocrine system, and other microenvironments, eventually leading to body damage, forming a fear of stress injury. Fear and anxiety, as a common psychological pressure in social groups, affects the normal life and work of patients by affecting the cognitive function of the brain and the mechanism of microenvironment. Therefore, in recent years, scientists at home and abroad have been devoted to exploring the mechanism of fear, in order to find out the impact of children on the immune system in the case of acute psychological stress and behavioral stress, and conduct a meta-analysis based on a large amount of data to find out the cause of the disease and targeted treatment to eliminate the impact of the disease. The research mainly focuses on the following aspects: the influence of fear on knowledge, the memory regression mechanism of fear, and the influence of fear on the immune system. A meta-analysis based on the study of children's acute psychological stress and behavioral stress on immune function under the microscope can be very effective in treating children's acute stress response and reducing psychological damage to children.

### 1.2. Innovation

The experiment uses a meta-analysis method to study the basic experiments of this method as a statistical method that combines the results of several independent studies with the same research objective for quantitative system evaluation. The second method is the inverse method of variation, also known as the weighted least squares method. This is the most common method after analysis. This method is based on the variability of research results. The relationship between the survey results was used as the total weight. The deviation is used to measure the degree of variance in a sample. The greater the variability, the greater the variability of the sample, and the less certainty the clustering parameter has, and the less the effect on the combined effect size. This method considers a fixed-effects model and a random-effects model. The simulation results show that this index has good statistical performance under various configurations.

The multiple data method was also used in the experiment. And the big data analysis framework created by this method is quite simple and efficient. At the same time, the parallel operation of multiple components is an attempt at a new approach to consolidating results. The majority of analytics surveys after many variables apply to the big data sector. The application of multivariate meta-analysis extends to the field of medical analysis, and the theory of multivariate meta-analysis has been developed. This is a method after multivariate analysis. To demonstrate the effect of this method, a sample of analysis and simulation experiments will be used together and selected multiple indicators to compare results. This makes the evaluation results more comprehensive and reliable.

### 1.3. Paper Organization

In this thesis, a meta-analysis is conducted on the impact of children's acute psychological stress and behavioral stress on immune function, and the whole process is related to observation under the microscope. The beginning of the thesis is to introduce the specific analysis of children's psychological conditions, the resulting psychological stress, and behavioral stress behavior, and finally lead to the impact on the immune function. After citing the research of several experts, it is found that a meta-analysis of the disease is carried out. Find out the reasons that affect immune function. In the method part, it analyzes the meta-analysis method, the risk assessment of deviation, the variance component model, and the multiple linear regression model, and has been applied in this article. In the experimental part, experiments were conducted on mice, and it was found that there were corresponding symptoms in the clinic to reflect the reasons for the impact of the patient's immune function. In the final discussion and summary part, using the results of clinical experiments in mice, it is concluded that acute psychological stress has an inhibitory effect on the immune function of the body and that proper load exercise cannot improve the immune function of the body.

## 2. Related Work

Exposure to stress results in physiological changes known as “stress response,” which are the result of changes in the activity of the adrenal medullary hormone system, hypothalamus pituitary adrenal (HPA), and sympathetic nervous system (SNS). Rakhshan studied the effects of chronic physiological and psychological stress on ischemia/reperfusion (I/R) injury in isolated rat hearts and the role of the sympathetic nervous system in stress. The rat hearts were isolated and subjected to ischemia for 30 min and reperfusion for 120 min. Daily stress was induced one week before I/*R* induction. Sympathectomy is accomplished by injecting hydroxydopamine before stress induction. There were no significant changes in heart rate and coronary flow between the two groups. The left ventricular diastolic blood pressure (LVDP) and rate overstock (RPP) in the physiological stress group and the psychological stress group were significantly lower than those in the control group (*P* < 0.05), but there was no significant difference between the physiological stress group and the psychological stress group [1, 2].

Psychogenic fever is a psychosomatic disease related to stress, especially in young women. Some patients have extremely high core body temperature (TC) (up to 41°C) when affected by emotional events, while others show persistent low-grade hyperthermia (37–38°C) under chronic stress. The mechanism of psychogenic fever is not fully understood. However, clinical case reports show that psychogenic fever is alleviated not only by antipyretic drugs, but also by psychotropic drugs showing anti-anxiety and sedative effects, or by natural means or psychotherapy to solve patients' difficulties. Oka studies have shown that psychological stress increases TC through a mechanism different from infectious fever (requiring proinflammatory mediators), and the sympathetic nervous system, especially the nonshivering heat production in brown adipose tissue mediated by *β*3-adrenoceptor, plays an important role in the occurrence and development of psychological stress-induced high fever [3, 4].

The mechanism of stress inflammation leading to severe depressive disorder remains unclear. AMI studied the role of adenosine triphosphate (ATP)/purinergic 2 × 7 receptor (P2X7R) pathway and NLRP3 (nucleotide binding, leucine-rich repeats, containing three pyrimidine domains) inflammatory bodies in interleukin-1*ß* (IL-1*β*) and stress-induced depressive behavior. The effects of acute restraint stress on extracellular ATP, glutamate, IL-1*ß,* and tumor necrosis factor-*α* in hippocampus were measured by microdialysis, and the effects of acute restraint stress on NLRP3 inflammatory bodies were analyzed by Western blot. In the chronic unpredictable stress model, the effects of P2X7R antagonist on IL-1*β*, tumor necrosis factor *α*, anxiety, and depression behavior were observed [5].

## 3. Mathematical Basis

### 3.1. Multivariate Meta-Analysis

In many scientific research directions, in the discussion of similar problems, different researchers will adopt the same or different mathematical theoretical methods for research and experiment, but the conclusions drawn from the experimental results are indeed similar. In the current situation, we discuss and summarize different research results, and finally come to a conclusion [6]. This problem can be solved by using a meta-analysis, which provides quantitative average results for the answers. In order to improve the accuracy of the conclusion, we need to increase the number of samples, collect more samples to explore the experiment, and effectively solve the problem of different experimental results. This is a quantitative review of the literature. It accepts the same results of several independent studies as the subjects [7]. In the implementation of strict research experiments, it is necessary to use good statistical methods to analyze and study the collected data, and to conduct an objective and quantitative comprehensive analysis of multiple research results.  Figure 1 shows the specific workflow of Mate's analysis.

A meta-analysis is a statistical method used to compare and synthesize the results of studies on the same scientific question. Whether the conclusion is meaningful depends on the quality of the included studies and is often used for quantitative pooled analysis in systematic reviews. In the use of a meta-analysis, we must first determine the impact value of the results, which can be used to measure the quality of research results, such as correlation coefficient, relative ratio, and standard relative deviation, which can be used as the effect value. The fixed result value is the basis of postanalysis. Only in the reliable comprehensive analysis of the results can we make a reliable comprehensive analysis of the results. In practical research, more than one effect value is often needed to evaluate the experimental or research results. For example, in terms of work, the evaluation of an employee's daily work performance is not only based on the employee's completion of the work, but also on the employee's performance in other aspects, such as attendance, coworkers' relationship, and work completion quality [8]. In the medical field, heart disease drug testing is to measure blood pressure when the heart is contracting, and it is also necessary to measure blood pressure in the process of expansion; in the financial field, there are many indicators reflecting the liquidity risk of enterprises, such as liquidity indicators, quick ratio, and short-term multiple cash liabilities. When summarizing the above research results, many researchers will choose to conduct a meta-analysis on each result value and then summarize the results as the overall evaluation [9, 10]. However, for the same population, there is often a correlation between different impact values. If each result value is regarded as an independent individual and analyzed separately, the correlation between each result value will be ignored, which may lead to overestimation of the change of effect value, and the estimation value of effect value is biased. The multivariate meta-analysis solves the problem that the unit meta-analysis ignores the correlation of evaluation indicators when analyzing multiple effect values, making the evaluation results more accurate. In addition, compared with individual unit meta-analysis, multivariate meta-analysis takes into account the correlation between impact values and can get more effective conclusions. Therefore, this analysis method can provide more accurate conclusions or reduce errors when some studies lack effect values or there are some unavoidable reference deviations.

### 3.2. Risk Assessment of Bias

The research and implementation of systematic evaluation and meta-analysis have been widely used in the medical field, especially the increase of randomized controlled trials and evidence-based medicine in recent years [11]. Researchers also regularly evaluate the quality of systematic reviews and meta-analysis studies. The schematic diagram of the researchers studying the immune function of young children is shown in Figure 2.

Multivariate analysis is a set of statistical theories and methods to study the relationship between multiple independent variables and dependent variables. Meta-analysis is a method of collecting data for quantitative and systematic evaluation. The quality of its conclusions depends not only on the preciseness of the postanalysis process, but also on the quality of the research literature itself and the reasonable control of deviation. Jada scale is also commonly used to analyze the quality of randomized controlled trials in a meta-analysis. Cochrane's participation in risk assessment tool has seven elements in six aspects of participation in risk assessment:

1. Selection: including random sequence generation and allocation hiding.
2. Implementation: including blinding of researchers and subjects.
3. Measurement: blind evaluation of study outcome.
4. Follow-up: research results of outcome data.
5. Report: selective report of research results.
6. Others: the origin of other biases.

According to the risk assessment criteria of bias, we made “low-risk bias,” “high-risk bias,” and “unclear.” Cochrane embedded software contains risk assessment tools and provides risk-sharing assessment results' chart, and colors such as green, red, and yellow can be selected and also symbols such as “+,”“-,” and “?” were “low-risk bias,” “high-risk bias,” and “unclear.”

Selection bias mainly involves three items: allocation sequence, baseline characteristics, and hidden grouping. However, with the release of the cyclone tool, the “low-risk” coincidence rate of the published animal experiments in these three items has been improved to some extent, but the actual proportion is less than 39%, of which the distribution sequence is only 12.74%, and the hidden grouping is less than 3%. Compared with clinical trials, the sample size of most animal experiments is small, and “random allocation” is not the standard practice mode in animal experimental research. Therefore, differences in some important baseline characteristics of animals between groups are more likely to affect the inference of experimental results. Moreover, randomization without hidden grouping still exaggerates the therapeutic effect. Therefore, we should pay more attention to the influence of baseline characteristics on the experimental results in future experiments, especially for the studies that have not been randomized or the sample size is relatively small. In addition, more attention should be paid to the implementation and development of random method and hidden grouping method in animal experimental research to reduce the selective bias.

### 3.3. Variance Component Model

The variance component model is a general term for both “random-effects model” and “mixed-effects model.” Meta-analysis is a combination of multiple studies (hypothesis K) on the same problem. In the idea of selection equation, a variable model is used to conduct statistical treatment on a meta-analysis. The basic idea is to treat the problems studied by a meta-analysis as a distributed population [12]. The results of the first study are samples taken from the population. Since a meta-analysis is vulnerable to the risk of heterogeneity and bias, the following two are used to describe the idea of modeling meta-analysis in the selection equation [13].

#### 3.3.1. Steady-State Model

The steady-state model shows that each study is homogeneous, and there is only one true effect value in each study time; that is, there is no difference between these studies. The difference of effect value directly observed from the study comes from the sampling error. The mathematical model is as follows:

(1) $$\begin{array}{c} y_{i}=\mu +\sigma_{i}\varepsilon_{i},\varepsilon_{i}∼N\left(0,1\right),\\ L\left(\beta |X,y\right)=\prod_{i=1}^{n}{\left[\pi \left(X_{i}\right)\right]}^{y_{i}}{\left[1-\pi \left(X_{i}\right)\right]}^{1-y_{i}}, \end{array}$$

where *y*_i_ is the estimated value of the effect value of the ith study, *µ* is the comprehensive effect value, and *σ*_i_^2^ is the variance of sampling in the population.

#### 3.3.2. Random-Effects Model

The random-effects model means that the actual impact value of each study is different, and the value of each study is subject to normal distribution. Therefore, the difference should include the random error and sampling error in the actual result value in the final audit. The mathematical model is as follows:

(2) $$\begin{array}{c} y_{i}=\mu_{i}+\sigma_{i}\varepsilon_{i},\mu_{i}∼N\left(\mu ,\tau^{2}\right),\varepsilon_{i}∼N\left(0,1\right),\\ l\left(\beta \right)=\sum_{i=1}^{n}\left\{y_{i}\ln\left[\pi \left(X_{i}\right)\right]+\left(1-y_{i}\right)\left[1-\pi \left(X_{i}\right)\right]\right\}. \end{array}$$

where *y*_i_ is the estimated value of the effect value of the ith study, *µ* is the comprehensive effect value, *t*^2^ is the variance between groups, *t* 2s used to measure the heterogeneity among groups of studies, and *σ*_i_^2^ is the variance of intragroup sampling.

### 3.4. Multiple Linear Regression Model

One of the most common statistical models is multiple linear regression model, which is widely used in various fields. Through multiple linear regression model, the correlation between independent variable and dependent variable can be obtained, or dependent variable can be predicted through independent variable [14]. Under normal circumstances, a multiple linear regression model with multiple independent variables can be written as follows:

(3) $$\begin{array}{c} y_{i}=\beta_{0}+\beta_{1}x_{1i}+\beta_{2}x_{2i}+\beta_{3}x_{3i}+\cdots +\beta_{k}xk_{1i}+u_{i},\;i=1,2,3,\ldots ,n, \end{array}$$

where *x* is the explanatory variable or independent variable and *β* is the correlation coefficient of each explanatory variable. Therefore, a multiple linear regression model is selected for the simulation experiment. The multiple regression model selected for the experiment is the quaternion regression model, and the model format is as follows:

(4) $$\begin{array}{c} y=\beta_{0}+\beta_{1}x_{1}+\beta_{2}x_{2}+\beta_{3}x_{3}+\beta_{4}x_{4}+\varepsilon , \end{array}$$

where *y* is the dependent variable, x_1_-x_4_ is the independent variable, *β*_0_-*β*_4_ is the five parameters of the model, and *e* is the random error term of the model. The variables of each model are sampled many times, and finally, multiple datasets are obtained. After receiving the data required by the simulation experiment, the data set is randomly divided into N parts for comparative analysis. After that, the simple average method and multivariate meta-analysis method were selected, and combined with the parameter estimation of N data items, the multivariate analysis model was established [15, 16].

Define how many positive packets at a certain point are close to the point and how far the point is from the negative packet example as the diversity density of the point. The probability of diversity density is expressed as follows:

(5) $$\begin{array}{c} y\left(x\right)=\text{ROOT}\left(x=t|C_{1}^{+},\ldots ,C_{n}^{+},C_{1}^{-},\ldots ,C_{m}^{-}\right), \end{array}$$

where *x* represents an independent point in the feature space, and *t* represents a factual concept. As such, the goal of the problem is to determine by maximizing the diversity density, namely,

(6) $$\begin{array}{c} \arg\underset{x}{\min}\text{ROOT}\left(x=t|C_{1}^{+},\ldots ,C_{n}^{+},C_{1}^{-},\ldots ,C_{m}^{-}\right),\\ \arg\underset{x}{\min}\prod_{i}\text{ROOT}\left(x=t|C_{i}^{+}\right)\prod_{i}\text{ROOT}\left(x=t|C_{i}^{-}\right). \end{array}$$

For positive or negative packets, the meaning of independent point *x* as a fact concept is also different. Assuming that the event only occurs if there is at least one cause for the event, the mathematical description of the model is as follows:

(7) $$\begin{array}{c} \text{ROOT}\left(x=t|C_{i}^{+}\right)=1-\prod_{j}\left(1-\text{ROOT}\left(x=t|C_{ij}^{+}\right)\right),\\ \text{ROOT}\left(x=t|C_{i}^{-}\right)=\prod_{j}\left(1-\text{ROOT}\left(x=t|C_{ij}^{-}\right)\right). \end{array}$$

The probability of an example appearing on a potential target is defined as the distance between the example and the potential target.

(8) $$\begin{array}{c} ROOT\left(x=t|C_{ij}\right)=\left(-{\left\|C_{ij}-x\right\|}^{2}\right),\\ {\left\|C_{ij}-x\right\|}^{2}=\sum_{n}S_{n}{\left(C_{ijn}-x_{n}\right)}^{2}, \end{array}$$

where *B*_*ijn*_ represents the *n* attribute of *B*_*ij*_, and *s*_*n*_ represents the correlation degree of the *n* attribute. In the logistic regression model, if the value of *y*_*i*_ is [0, 1], then

(9) $$\begin{array}{c} P\left(y_{i}=1|M_{i}=m_{i}\right)=\gamma \left(m_{i}^{\prime }\varepsilon \right),\\ \gamma \left(x\right)=\frac{\exp\left(x\right)}{1+\exp\left(x\right)}={\left(1+\exp\left(-x\right)\right)}^{-1}. \end{array}$$

The parameter likelihood function of *ε* is

(10) $$\begin{array}{c} \text{ROOT}=\prod_{i=1}^{n}{\left[\gamma \left(m_{i}^{\prime }\varepsilon \right)\right]}^{y_{i}}{\left[1-\gamma \left(m_{i}^{\prime }\varepsilon \right)\right]}^{1-y_{i}},\\ \text{ROOT}=\sum_{i=1}^{n}y_{i}\log\;\gamma \left(m_{i}^{T}\varepsilon \right)+\left(1-y_{i}\right)\log\left[1-\gamma \left(m_{i}^{T}\varepsilon \right)\right]. \end{array}$$

The estimated variance can be obtained after derivation of the above formula with respect to parameter *ε*

(11) $$\begin{array}{c} \sum_{i=1}^{n}\left(\frac{y_{i}}{\gamma \left(m_{i}^{T}\varepsilon \right)}-\frac{1-y_{i}}{1-\gamma \left(m_{i}^{T}\varepsilon \right)}\right)\gamma^{\prime \prime }\left(m_{i}^{T}\varepsilon \right)m_{i}=0. \end{array}$$

By this, *γ*^″^(*x*) means

(12) $$\begin{array}{c} \frac{\text{d}}{\text{d}x}\gamma^{\prime \prime }\left(x\right)=\frac{\exp\left(-x\right)}{{\left(1+\exp\left(-x\right)\right)}^{2}}=\gamma^{\prime \prime }\left(x\right)\left(1-\gamma^{\prime \prime }\left(x\right)\right). \end{array}$$

After calculation, the estimation equation can be simplified to

(13) $$\begin{array}{c} \sum_{i=1}^{n}m_{i}\left(y_{i}-\gamma \left(m_{i}^{T}\varepsilon \right)\right)=0. \end{array}$$

## 4. Experimental Design and Analysis

Machine learning is a multifield interdisciplinary subject involving probability theory, statistics, approximation theory, convex analysis, algorithm complexity theory, and other disciplines. It specializes in how computers simulate or realize human learning behaviors to acquire new knowledge or skills, and to reorganize existing knowledge structures to continuously improve their performance. Deep learning is to learn the inherent laws and representation levels of sample data, and the information obtained during these learning processes is of great help to the interpretation of data such as text, images, and sounds. Its ultimate goal is to enable machines to have the ability to analyze and learn like humans, and to recognize data such as words, images, and sounds. Deep learning is a complex machine learning algorithm that has achieved results in speech and image recognition far exceeding previous related technologies.

### 4.1. Experimental Animals

The rats used in the experiment are provided by Beijing Siberian Experimental Animal Co., Ltd., which are closed group, clean grade, and have license number identification. The animal rearing environment is in line with the relevant ethical requirements of animal experimental research.

### 4.2. Experimental Methods

Fifteen male rats, aged about 5 years old and weighing about 250g, were reared adaptively for 10 days in the environment of relative humidity 70%, illumination time 8 : 00–18 : 00, and temperature about 25°C. The experiment began one week later. Male rats were randomly divided into three groups: placebo control group, placebo stress group, and drug stress group, with 5 rats in each group. The placebo control group ate and drank normally without stress. The stress patterns of placebo stress group were fasting for one day, water deprivation for 8 hours, empty bottle stimulation for 3 hours, tail stimulation for 10 minutes, strange object stimulation for 8 hours, and immobilization for 3 hours. In addition to the above three different stress modes daily for 5 consecutive weeks in the fasting stress group, the same stress mode should not persist. 3 ml/D (5 mg/kg) of 0.7% normal saline and 4 ml/D (5 mg/kg) of hydrogen bromide solution were injected subcutaneously. The preference rate of sugar water = sugar water intake/total intake × 100% was calculated according to the preference degree of sugar water. Sugar preference was calculated before the beginning of stress stimulation, at the end of the second and third weeks. The rats were randomly divided into a control group, a chronic stress group, and a chronic pain group. The technical route is shown in Figure 3.

### 4.3. Quality Control

It is necessary to strictly control the quality of each step. All personnel involved in the research should be trained uniformly to ensure homogeneity. In the process of the experiment, it needs to be completed on time according to the planned research method. The problems encountered in the experiment need to be dealt with in time and the research scheme should be improved. When recording the data, the trained team members should be unified to input the data, and the two people should check the data to ensure the authenticity and accuracy of the data to the maximum extent.

### 4.4. Statistical Methods

The software was used to conduct a meta-analysis on the data, and the related risk and its 93% confidence interval were selected as the results of binary variables. If the variable is continuous variable, the standard mean deviation and weighted average deviation shall be adopted when the measurement method and unit are consistent. As a result of the inconsistency between measurement method and measurement unit, continuous variable index is combined with weighted average difference, and binary classification index is combined with RR. When *p* < 0.05, the changes of the results were considered to be statistically significant. Subgroup analysis of heterogeneity indicators was performed to obtain the sources of heterogeneity, and sensitivity analysis (exclusion) was used to evaluate the overall results of the study.

## 5. The Effect of Stress on Immune Function

### 5.1. Changes of Substances after Stress

The changes of substance levels in the body before and after the stress reaction can be seen from the figure that the level of leptin has a considerable change before and after the stress reaction. From the figure, the change of leptin plasma concentration in rats is described in the figure: after the implementation of stress response stimulation, the leptin level of rats decreased to 54% of the normal in the process, and then gradually increased. After one day of stress reaction, the level of leptin basically returned to the basic level; in the rats in the placebo stress group, the leptin level showed a similar change with the previous group, gradually recovered to 58% of the normal during the operation, and then showed a gradual recovery trend, as shown in Figure 4.

Cortisol level in the first group of rats increased significantly during the stress reaction, gradually decreased, and then decreased to the basic level in the day after the stress response. As part of cardiopulmonary bypass (CPB), the level of leptin and cortisol in rats was negatively correlated after in vitro stimulation. In the placebo stress group, the cortisol level gradually increased from the stress reaction to the middle of the day, peaked at two hours after the reaction, and then decreased, but the change of cortisol level was not statistically significant.

In the placebo control group, the level of IGF-1 increased significantly two hours after the stress reaction and then gradually decreased. It dropped to the basic level in one day after the reaction and decreased to a lower level after two days. There was a significant correlation between cortisol and IGF-1 levels. IGF-1 levels tended to be negatively correlated with leptin levels, but there was no significant difference between them. The changes of IGF-1 levels in the placebo stress group were similar to those in placebo control group.

### 5.2. Effect of Stress on Weight Gain

The weight gain of the control group and the experimental group during the 18-day restraint treatment was shown. Two-dimensional analysis of variance showed that there were significant differences in restraint, time, and the interaction between constraint and time. At the beginning of chronic restraint, there was no significant difference in body weight between the two groups, but the weight gain of rats in the experimental group was significantly slowed down from the fifth day. This result shows that our chronic restraint treatment can effectively induce chronic stress response in rats, as shown in Figure 5.

It can be seen from the figure that the weight gain of the control group is higher than that of the stress response group, and the weight jump-like growth appears on the ninth day. Although the difference of weight growth rate between the two experimental groups was not significant in the first six days, the difference of weight change rate was bigger with the increase of time. The weight of stress response group began to increase steadily on the 15th day.

### 5.3. Sugar Preference

Sugar water preference test was used to test the level of pleasure loss. The behavioral results of rats in this study showed that compared with the drug stress group and the placebo control group, the placebo stress group had less basic fine action, longer resting time, and lower preference for sugar solution, which indicated that chronic stress led to depression-like behavior, increased tension, decreased interest, and cognitive function of exploration. It is similar to fatigue, energy decline, psychomotor depression, and interest decline in patients with depression.

After three weeks of chronic unpredictable mild stimulation and control group mice, their emotional state was evaluated by sugar water preference test. Depressive behaviors were as follows: after chronic unpredictable mild stimulation, the consumption of sugar water was significantly lower than that before chronic unpredictable mild stimulation; the exploration time of new things after chronic unpredictable mild stimulation was significantly lower than that before chronic unpredictable mild stimulation. If the mice showed significant changes in this experiment, they were defined as chronic unpredictable mild stimulation-induced depression-like mice, and if the mice did not show significant changes in the three experiments, they were defined as chronic stress resistance mice, as shown in Figure 6.

The preference of sugar water is expressed by SPT value, SPT value = sugar water amount/(sugar water amount + pure water amount) × 100%. The first group of histograms shows the changes of SPT values before and after chronic unpredictable mild stimulation in depression-like mice induced by chronic unpredictable mild stimulation; the second group shows the changes of SPT values in chronic unpredictable mild stimulation of the chronic stress resistance group; the third group shows the changes of SPT values of control group mice in the same period. Chronic unpredictable mild stimulation resulted in a significant decrease in sugar preference in depression-like mice, but no significant change was observed in the chronic stress resistance group.

It can be seen from the figure that the SPT value of depression-like mice induced by chronic unpredictable mild stimulation was 94% before chronic unpredictable mild stimulation and 63% after chronic unpredictable mild stimulation, while the SPT value of mice in the chronic stress resistance group was 93% before chronic unpredictable mild stimulation and 92% after chronic unpredictable mild stimulation. Meanwhile, the SPT values of the control group were 94% and 93%, respectively, before and after the experiment. The results showed that the depression-like mice induced by chronic unpredictable mild stimulation showed a significant decrease in sugar water preference, while the mice in the chronic stress resistance group after chronic unpredictable mild stimulation did not change significantly.

### 5.4. Proportion of T Lymphocyte Subsets

After the experimental operation, 1 ml venous blood was drawn from rats on an empty stomach. The peripheral blood mononuclear cells were extracted by density gradient centrifugation. The proportion of T lymphocyte subsets (CD4 +, CD8 + and CD4 + /CD8 +) was detected by Beckman flow cytometry. The results showed that the proportion of CD4 + T lymphocytes increased in thymopentin group and Bozhi glycopeptide group compared with the placebo group, the difference was statistically significant, and there was no significant difference in CD8 + T lymphocyte among the three groups. CD4 + /CD8 + represents the ratio of *T* helper cells/*T* suppressor cells, referred to as CD4 + /CD8 +. The results showed that after 3 weeks of experiment, the ratio of CD4 + /CD8 + in thymopentin group and Bozhi glycopeptide group was higher than that in the placebo group, and the difference was statistically significant. Flow cytometry was used to detect the proportion of T lymphocyte subsets in human peripheral blood. The specific situation is shown in Figure 7.

After drug injection, the proportion of peripheral blood T lymphocytes was detected by flow cytometry. The statistical results showed that compared with the placebo group, the difference of CD4 + in thymopentin group and Bozhi glycopeptide group was statistically significant, but the difference of CD8 + was not statistically significant.

### 5.5. The Effect of High-Intensity Exercise and Acute Psychological Stress on Behavior and Weight

#### 5.5.1. Subjects and Feeding

The animals adapt to the laboratory environment for a week, during which they are stroked irregularly and for a short period of time every day to reduce the impact of the operation. At the same time, the high-intensity exercise group was placed on the animal treadmill for training every day, and the entire experimental period lasted for seven weeks. The weight comparison between rats in each group is shown in Table 1.

#### 5.5.2. Dynamic Observation of Rat Behavior

The rats in the quiet control group were in good condition, with normal daily food intake, bright coat color, standing on the two legs of the box wall, many searching movements, and gentle temperament. The hair color of rats in the high-intensity exercise plus chronic psychological stress group is yellowish. With the continuation of exercise and psychological stress, the food intake gradually decreases, especially in the last week of the experiment, and the food intake per day is only equivalent to one meal in the quiet control group. The food intake and weight changes of rats in each group are shown in Figure 8.

It can be seen from Figure 8 that the rats in the quiet control group have been gaining weight steadily, followed by the rats in the chronic psychological stress group; the rats in the high-intensity exercise plus chronic psychological stress group have the smallest increase in weight; and the rats in the high-intensity exercise group have the smallest increase in weight between the latter two.

#### 5.5.3. Results of Determination of Blood Urea Nitrogen Content

It can be seen from Table 2 that the high-intensity exercise plus chronic psychological stress group had higher blood urea nitrogen levels after exercise and psychological stress than in the psychological stress group (*P* < 0.05) and the quiet control group (*P* < 0.01); the blood urea nitrogen level at 24h after stress decreased significantly (*P* < 0.05); and the blood urea nitrogen level at 24h after psychological stress was much lower than that of the quiet control group (*P* < 0.01).

#### 5.5.4. White Blood Cell Count Result

The variance analysis of high-intensity exercise and acute psychological stress on white blood cells (WBC) of rats is shown in Table 3.

It can be seen from Table 3 that there is no significant difference between each group and the quiet control group. But at the moment of psychological stress, the number of WBCs in group P was significantly higher than that in EP and *E* groups (*P* < 0.05), and there was no significant difference between the latter two groups. The effects of high-intensity exercise and acute psychological stress on the thymus index and spleen index of rats are shown in Tables 4 and 5.

It can be seen from Table 4 that there is no significant difference in the thymus index between the groups after long-term high-intensity exercise and chronic psychological stress immediately and after 24 hours.

### 5.6. Effects of Drugs on Immune Function

The traditional Chinese medicine compound is composed of *Astragalus* membranaceus, radix rehmanniae, Codonopsis pilosula, and Angelica sinensis, which are fermented by *Saccharomyces cerevisiae* and *Bacillus* subtilis. All the herbs were purchased from Wuhan Hanrongda Chinese Herbal Medicine Co., Ltd. The main production process is as follows: first, the raw materials are processed, the processed traditional Chinese medicine is dried and crushed, and then, the auxiliary materials and microbial agents are added according to a certain formula, mixed evenly, and then bagged for use.

The changes of blood lymphocytes and white blood cells in rats are shown in Table 6. It can be seen that the number of all kinds of cells in the blood of the rats in the third group of the experiment was not significant. After the beginning of the experiment, the number of lymphocytes and white blood cells increased significantly with the increase of the amount of traditional Chinese medicine, especially on the 10th and 15th days of the experiment; the 50 and 75g/*D* groups were significantly higher than the control group; and the highest number of lymphocytes and white blood cells appeared in the 100g/*D* groups on the 15th day, 03 × 109/*L* and 1.97 × 109/*L*, respectively. At the same time, it was found that there was no significant difference in the number of blood granulocytes and white blood cells in all groups during the whole experimental period.

### 5.7. Effect of Different Load Exercise on IL-6 Content in Rats with Acute Psychological Stress

It can be seen from Table 7 and Figure 9 that the two-factor analysis of variance was used to test the effects of acute psychological stress and exercise on the IL-6 content of rats. The results showed that the analysis of the 10-minute exercise acute psychological stress (S1P1) group and minute exercise in the difference of IL-6 in P1 group, F = 5.613, *P* < 0.05, suggesting that the difference in IL-6 content between S1P1 group and S0P1 group is significant, and the IL-6 content of S1P1 group is higher than that of P1 group. Analyze the difference in IL-6 between the 60-minute exercise acute psychological stress (S1P2) group and the minute exercise (P2) group, *F* = 24.742, *P* < 0.01, suggesting that the IL-6 content difference between the S1P2 group and the P2 group is very significant sex, and the IL-6 content of S1P2 group was lower than that of P2 group. The results of experiments conducted through the above multiple methods show that these methods can be used clinically to conduct a meta-analysis of children's acute psychological stress and behavioral stress, and use a microscope to study and analyze the specific conditions of patients.

## 6. Conclusions

Stress response is a kind of physical defense. If the response to stress is very strong and takes a long time, it is harmful to the body, and often there will be pathological changes, known as the pathological response of stress, and this phenomenon is called general adaptation syndrome. Initially, stress refers to the biological response of human or animal organisms to environmental stimuli, which may be caused by many different requirements on the body, not specific. Stress refers to the environment or internal needs beyond the adaptability of individual, society or body organization system, or people have special physiological or psychological needs, and thus produce unusual or unexpected reactions. Stress response is a nonspecific defense response to harmful stimuli. This mechanism includes stimulation of sympathetic nerve and inhibition of sympathetic nerve. Effective control and interruption of stress response have a positive impact on the mechanism. The increase of catecholamine excretion caused by stress reaction can cause many cardiovascular reactions. Insulin secretion decreases, and glucose secretion increases. Catecholamine produced by stress reaction is an important factor in the development of tumor. Professor Rakhshan's research is aimed at the effects of chronic physiological and psychological stress on ischemia/reperfusion (I/R) injury of isolated rat hearts and the role of the sympathetic nervous system in stress, and there is no relevant change in the human body. Professor Oka's research shows that psychological stress increases TC through a mechanism different from infectious fever (which requires pro-inflammatory mediators) and the sympathetic nervous system. His research lacks the support of experimental data, so I do not want this experiment to do a lot of experiments.

This meta-analysis provides a reference for the characteristics of children's psychological acute stress. It is hoped that the research results can provide a possible research direction for clinicians in treating children's immune function impairment caused by stress reaction. This study only analyzes the cognitive effect of stress-induced simple graphics in rats, and the following research should analyze spatial knowledge and knowledge-related attention factors. Due to the limited number of relevant high-quality studies and the small sample size, the validity of the evidence in the conclusion is limited to a certain extent. Therefore, it is expected to have a higher quality, large sample multicenter study to further explore the efficacy of stress-induced immune damage. The medical image fusion research based on deep belief network introduces medical images in detail. In this article, the microscope observation experiment provides a large number of research methods, which makes the experiment very smooth, and deep neural network multimodal medical image based on multi-objective differential evolution. Fusion technology describes the application of deep neural networks in image fusion and provides a research direction for this article; the study of drug synergistic effect prediction based on dynamic mutation and differential evolution provides a good explanation of the synergistic effect of drugs. Different drugs are used to work together in one body, which can effectively illustrate the results of the experiment.

In order to carry out normal immune regulation, human body must have a complete and coordinated immune system composed of immune cells, immune cells and immune organs. The thymus and bone marrow of malignant gland and central immune organ are the mature sites of T lymphocyte and B lymphocyte, respectively. Spleen has the function of filtering blood and bleeding, but as the largest immune organ of human body, it is more for the maturation of various immune cells and when pathogenic bacteria invade the human body's fungi and cells. This study is to conduct a meta-analysis of the effects of children's acute psychological stress and behavioral stress on the immune function, and use a microscope to conduct specific observations on white mice. The experimental research results show that the evaluation of animal models and the study of the physiological mechanism of psychological disorders are of great significance. This research provides a reliable pressure model for the neural mechanisms and methods that express different degrees of fear in the subsequent visual pathways to transmit and receive sensory information.

## Figures and Tables

**Figure 1:** The specific workflow chart of a meta-analysis.

**Figure 2:** Schematic diagram of immune function.

**Figure 3:** Technology roadmap.

**Figure 4:** Changes of stress substance levels.

**Figure 5:** Weight gain rate.

**Figure 6:** Sugar preference.

**Figure 7:** Proportion of lymphocyte subsets.

**Figure 8:** Rat body weight change.

**Figure 9:** The effect of exercise on the content of IL-6 in rats with acute psychological stress.

**Table 1:** Weight comparison between rats in each group.

Group	Deal with	N	Weight(g)
EP1	High-intensity exercise plus psychological stress immediate group	8	200.32 ± 13.62
EP2	24-h group after high-intensity exercise plus psychological stress	8	208.17 ± 12.73
E3	High-intensity exercise immediate group	8	208.14 ± 17.33
E4	24-h group after intensive exercise	8	210.39 ± 11.47
P5	Chronic psychological stress immediate group	8	199.93 ± 20.56
P6	24-h group after chronic psychological stress	8	197.43 ± 14.56
C	Quiet control group	8	199.72 ± 13.26
Total	—	56	204.27 ± 15.67

**Table 2:** Comparison of blood urea nitrogen content.

Group	N	Blood urea nitrogen
EP1	7	188.32 ± 23.94
EP2	7	172.94 ± 19.33
E3	6	210.22 ± 30.62
E4	8	173.41 ± 41.27
P5	7	183.79 ± 24.09
P6	6	146.32 ± 24.71
C	7	207.32 ± 10.51

**Table 3:** Comparison of rat white blood cells (WBC).

Group	N	Blood urea nitrogen
EP1	7	7.36 ± 1.98
EP2	5	9.06 ± 2.13
E3	6	7.02 ± 1.24
E4	8	7.39 ± 2.18
P5	7	9.62 ± 1.26
P6	8	9.00 ± 3.40
C	7	8.90 ± 1.69

**Table 4:** Thymus index comparison.

Group	N	Blood urea nitrogen
EP	13	0.0013 ± 0.0005
E	14	0.0014 ± 0.0003
P	16	0.0012 ± 0.0003
C	7	0.0013 ± 0.0002

**Table 5:** Thymus index comparison.

Group	N	Blood urea nitrogen
EP	13	0.0028 ± 0.0008
E	14	0.0025 ± 0.0003
P	16	0.0029 ± 0.0004
C	7	0.0023 ± 0.0002

It can be seen from Table 5 that the spleen index of group P is much higher than that of group C and *E* (*P* < 0.01).

**Table 6:** Effects of drugs on immune function.

	0g/d	25 g/d	50 g/d	75 g/d	100 g/d
Granulocyte	3.41 × 10^9^/L	3.58 × 10^9^/L	3.82 × 10^9^/L	3.92 × 10^9^/L	4.01 × 10^9^/L
White blood cell	1.72 × 10^9^/L	1.83 × 10^9^/L	1.92 × 10^9^/L	1.84 × 10^9^/L	1.97 × 10^9^/L
Lymphocyte	2.45 × 10^9^/L	3.41 × 10^9^/L	3.89 × 10^9^/L	4.35 × 10^9^/L	5.03 × 10^9^/L

**Table 7:** Effects of different load exercises on the content of IL-6 in rats with acute mental stress.

	No exercise (P0)	30 minutes of exercise (P1)	60 minutes of exercise (P2)
Psychological stress (S1)	220.28 ± 72.21	452.17 ± 34.04	294.25 ± 82.11
No psychological stress (S0)	348.45 ± 63.54	429.12 ± 54.02	464.36 ± 97.19

## Data Availability

The data that support the findings of this study are available from the corresponding author upon reasonable request.
